The article "A Study on Risk Factors Associated with Reflux Esophagitis in Patients Undergoing Esophageal Cancer Surgery" was retracted in 2023. Reason: concerns about the peer review.

# A Study on Risk Factors Associated with Reflux Esophagitis in Patients Undergoing Esophageal Cancer Surgery

**DOI:** 10.1155/2022/3409693

**Published:** 2022-03-27

**Authors:** Ping Wang, Chunzhi Liu, Lianmin Wei, Wenchao Wei, Zhao Liu, Fengting Wu, Rui Qu

**Affiliations:** ^1^Department of Gastroenterology, Peoples' Hospital of Dongying, Dongying 257091, Shandong Province, China; ^2^Burn and Plastic Surgery, Shengli Oilfield Central Hospital, Dongying 257100, Shandong Province, China

## Abstract

**Objective:**

To investigate the risk factors associated with reflux esophagitis in patients undergoing esophageal cancer surgery and to provide reference for the prevention and treatment of reflux esophagitis.

**Methods:**

In the manner retrospective study, the data of 300 patients with esophageal cancer who received the surgical treatment in our hospital (January 2018–December 2020) were retrospectively reviewed. The 300 patients were divided into the occurrence group (*n* = 45) and nonoccurrence group (*n* = 255) depending on whether they had reflux esophagitis after surgery. The social demographic data and clinical data of the patients in the two groups were collected. These data were classified into the personal factors and surgical factors. The single-factor analysis method was adopted to analyze the effects of the personal and surgical factors on reflux esophagitis. The factors with statistically significant differences in the single-factor analysis were analyzed by logistic regression to verify the factors were the risk factors associated with reflux esophagitis in patients undergoing esophageal cancer surgery.

**Results:**

The differences in the bodyweight, body mass index (BMI), length of the resected esophagus, surgical approach, intraoperative blood loss, gastrointestinal decompression volume, and surgery time between the two groups were of statistical significance (*P* < 0.05). After being tested by the logistics multivariate analysis, length of the resected esophagus, whole stomach reconstruction, intraoperative blood loss, and surgery time were identified as the risk factors associated with reflux esophagitis in patients undergoing esophageal cancer surgery.

**Conclusion:**

The length of the resected esophagus, whole stomach reconstruction, intraoperative blood loss, and surgery time were the risk factors associated with reflux esophagitis in patients undergoing esophageal cancer surgery. It is necessary to choose the appropriate surgical approach according to the patients' conditions in practice and to strengthen the prevention and treatment of reflux esophagitis.

## 1. Introduction

Esophageal cancer, as a kind of malignant tumor originating from the esophageal epithelium, features strong invasion and high malignant degree. According to the International Agency for Research on Cancer under the World Health Organization, there were 572000 new patients with esophageal cancer worldwide in 2018 and 509000 patients died in the same year [1, 2]. In China, the incidence of esophageal cancer is high, and the yearly new and dead patients with esophageal cancer account for more than half of the global total [3]. Because the patents with esophageal cancer have no specific symptom at the early stage, most patients, with late diagnoses and poor prognoses, can only be treated with individualized comprehensive treatment centering on surgical treatment. Surgery is an important way to enhance the survival rate of the patients. In clinics, the stomach is generally used as a substitute to connect the esophageal stump, so as to guarantee the patients' digestive system function, but reconstruction of the esophagus with the stomach inevitably destroys the lower esophageal sphincter and other mechanical reflux barriers [4], so the patients are likely to develop the symptom of gastroesophageal reflux after surgery. Gastroesophageal reflux refers to the reflux of the contents in the stomach and duodenum into the esophagus, and the inflammatory lesion caused by it is called as reflux esophagitis [5]. Reflux esophagitis is the most common secondary disorder of gastrointestinal motility after esophageal cancer surgery. The patients with reflux esophagitis have different degrees of heartburn, abdominal pain, indigestion, and other symptoms, and even severe vomiting and dyspnea in severe cases, impacting their postoperative quality of life [6, 7]. According to the report of Bevilacqua et al., because the long-term reflux stimulation aggravates the metaplasia of esophageal mucosal tissues, the reflux esophagitis increases the possibility of the recurrence of esophageal cancer after surgery [8]. Investigating the risk factors associated with reflux esophagitis in patients undergoing esophageal cancer surgery is conducive to the prevention and treatment of reflux esophagitis, so as to ensure the patients' quality of life. Based on the retrospective analysis of 300 patients with esophageal cancer who received the surgical treatment, this study explores the relations between the occurrence of reflux esophagitis and the personal and surgical factors, attempting to provide clinical reference.

## 2. Materials and Methods

### 2.1. General Data

The data of 300 patients with esophageal cancer who were treated in our hospital (January 2018–December 2020) were retrospectively reviewed. Among 300 patients, 120 patients had the symptoms of retrosternal discomfort, burning sensation, and dragging pain, 164 patients had different degrees of dysphagia, throat pain, and hoarseness, and 16 patients had no symptom and found the esophageal cancer through gastroscopy or other examinations. All the patients were diagnosed as esophageal cancer by biopsy or pathological examination of surgical specimens and received the surgical treatment [9]. They were divided into the occurrence group (*n* = 45) and nonoccurrence group (*n* = 255) depending on whether they had reflux esophagitis after surgery. In the occurrence group, there were 32 males and 13 females with the mean age of (59.36 ± 5.27) years old. In terms of the histological type, there were 30 cases with squamous cell carcinoma, 12 cases with adenocarcinoma, and 3 cases with undifferentiated carcinoma. In the nonoccurrence group, there were 185 males and 70 females with the mean age of (59.31 ± 5.19) years old. In terms of the histological type, there were 162 cases with squamous cell carcinoma, 73 cases with adenocarcinoma, and 20 cases with undifferentiated carcinoma.

### 2.2. Diagnostic Criteria

All the patients received the barium meal radiography and gastroscopy and met the diagnostic criteria for reflux esophagitis. The patients had hiccough, nausea, and vomiting bile. The patients had bitter taste or manifestation of chronic laryngitis. The patients' gastroscopy showed that the digestive juice reversely flowed into the esophagus, and hyperemia and edema occurred in the median and lower esophagus and the mucosa of anastomotic orifice. The patients had the symptom of reflux when taking the erect position with the forward tilt angle of 30° in the barium meal radiography.

### 2.3. Moral Consideration

This study conformed with the principle of Declaration of Helsinki (2013) [10], and the patients had signed the informed consent.

### 2.4. Analysis Method

The social demographic data (sex, age, bodyweight, and body mass index (BMI)) and clinical data (tumor stage, histological type, tumor location, and surgical condition) of the patients in the two groups were statistically analyzed, and these data were classified into the personal factors and surgical factors. The personal factors included the sex, age, bodyweight, body mass index (BMI), tumor stage, histological type, and tumor location. The surgical factors included the length of the resected esophagus, gastric tube/whole stomach reconstruction, surgery time, intraoperative blood loss, days of gastrointestinal decompression, and gastrointestinal decompression volume.

### 2.5. Statistical Treatment

The software SPSS 20.0 was adopted to process the data. The univariate analysis of the patients' personal factors and surgical factors was conducted by using the *X*^2^ test and *t*-test, and the variables with *P* < 0.05 in the univariate analysis were included in the logistics regression model to conduct multivariate analysis. When *P* < 0.05, the differences were considered statistically significant.

## 3. Results

### 3.1. Univariate Analysis

The differences in bodyweight, BMI, resected length of esophagus, surgical approach, intraoperative blood loss, gastrointestinal decompression volume, and surgery time between the two groups were of statistical significance (*P* < 0.05; Tables 1 and 2).

### 3.2. Multivariate Analysis

After being tested by the logistics multivariate analysis, the length of the resected esophagus, whole stomach reconstruction, intraoperative blood loss, and surgery time were identified as the risk factors associated with reflux esophagitis in patients undergoing esophageal cancer surgery (Table 3).

## 4. Discussion

Reflux esophagitis, as the most common secondary disorder of gastrointestinal motility after the esophageal cancer surgery, refers to the inflammatory lesions caused by the reflux of the contents in the stomach and duodenum into the esophagus [11]. According to the survey by scholar Liu Xiao-Long, 8.90% of the residents in Beijing and Shanghai have the symptom of gastroesophageal reflux in different degrees, and the actual probability of developing gastroesophageal reflux disease is 5.70%. Among these patients, about 33.3% suffer from reflux esophagitis [12]. Among patients undergoing esophageal cancer radical surgery, the incidence of reflux esophagitis is higher. According to the report of Nejat Pish-Kenari Fatemeh et al., the incidence of reflux esophagitis in patients undergoing esophageal cancer surgery is 13.7%, indicating that surgery is the direct cause of reflux esophagitis [13]. Under normal conditions, the flake-like flapper effect of the lower esophageal sphincter and esophagogastric angle and the “spring clip” effect of the esophageal opening jointly form the antireflux mechanism. However, the esophageal cancer surgery negatively affects the antireflux mechanism because this treatment uses the stomach to replace the esophagus, completely destroying the integrity and anatomic structure of the esophagus [14, 15]. This treatment places the stomach in the negative-pressure thoracic cavity, which increases the gastric tension and volume, and the breathing, cough with asthma, and abdominal pressure all affect the gastroesophageal pressure to varying degrees, allowing gastric contents to flow into the esophageal lumen. Besides, the surgery severs the vagus trunk and damages the patients' autonomic nerve. The reconstructed neurological function of alimentary canal losses rhythmicity and naturality [16, 17], causing the delayed gastric emptying. As a result, the pylorospasm leads to the gastric outlet obstruction, bringing about gastrectasia and gastric retention, which aggravates the gastroesophageal reflux to some extent [18, 19]. Among 300 patients in this study, there were 45 patients having reflux esophagitis (including symptomatic reflux and pathological reflux), with the total incidence of 15.0%. Comparing the data of the occurrence group and the nonoccurrence group, it can be seen that the differences in the bodyweight, BMI, resected length of the esophagus, surgical approach, intraoperative blood loss, gastrointestinal decompression volume, and surgery time between the two groups were of statistical significance (*P* < 0.05). After being tested by the logistics multivariate analysis, the length of the resected esophagus, whole stomach reconstruction, intraoperative blood loss, and surgery time were identified as the risk factors associated with reflux esophagitis in patients undergoing esophageal cancer surgery and were closely related to the occurrence of reflux esophagitis.

At present, the effects of the gastric tube and whole stomach reconstruction on the postoperative complications have been confirmed. Most studies have concluded that the gastric tube with narrow top and wide bottom is closer to the physiological structure of the esophagus and can minimize the changes of the thoracic cavity, so adopting the gastric tube can reduce the incidence of postoperative complications and improve the patients' quality of life [20, 21]. There is no final conclusion on whether the gastric tube can reduce the incidence of reflux esophagitis. According to scholars Manning et al., the gastric tube can reduce the retention of food in the stomach, thus avoiding the occurrence of reflux [22]. However, the study of scholars Yusaku et al. shows that the effects of the gastric tube on preventing gastroesophageal reflux after surgery is not satisfactory, and the incidence of reflux esophagitis in patients undergoing esophagectomy is 22.5% [23]. This study has found that the incidence of reflux esophagitis in patients undergoing gastric tube reconstruction is lower, and the reasons are as follows. In normal physiology, the gastric oxyntic gland mainly exists in the body and fundus of the stomach. After esophagectomy, the oxyntic gland cells are decreased and neuromodulation is impeded. Under this condition, the gastric tube can reduce the compression from cough and breath on the thoracic stomach, thus reducing the reflux time and reflux volume. In this way, the gastric tube prevents reflux esophagitis. The shorter resected esophagus means less change of the involved physiological structure [24], so it is speculated that the resected length of esophagus is an important factor in the occurrence of reflux esophagitis after surgery. Besides, this study has also found that intraoperative blood loss and surgery time are the risk factors associated with reflux esophagitis, and the reasons are as follows. The patients with prolonged surgery time often have more complex conditions, and the amount of intraoperative blood loss intensifies the fluctuation of blood flow and aggravates the perioperative stress response, which elevates the occurrence rate of complications. According to scholars Fabian et al., the occurrence rate of complications among the patients with shorter surgery time is lower [25], indicating the relationship between surgery time and postoperative complications. Therefore, it is necessary to choose the appropriate surgical approach according to the patients, and it is better to choose the gastric tube surgery. At the same time, the patients with longer surgery time should actively receive postoperative preventive measures to prevent the occurrence of reflux esophagitis.

In conclusion, the length of the resected esophagus, whole stomach reconstruction, intraoperative blood loss, and surgery time were the risk factors associated with reflux esophagitis in patients undergoing esophageal cancer surgery. It is necessary to choose the appropriate surgical approach according to the patients' conditions in practice and to strengthen the prevention and treatment of reflux esophagitis.

## Figures and Tables

**Table 1:** Analysis of the patients' personal factors.

Group	Occurrence group (*n* = 45)	Nonoccurrence group (*n* = 255)	*X* ^2^/*t*	*P*
Sex			0.040	0.842
Male	32	185		
Female	13	70		
Age (years old)	59.36 ± 5.27	59.31 ± 5.19	0.059	0.953
Bodyweight	60.11 ± 2.65	62.98 ± 2.47	7.107	<0.001
BMI (kg/m^2^)	21.66 ± 1.28	22.10 ± 1.32	2.071	0.039

Tumor stage				
T1N0M0	2	30	2.151	0.142
T2N0M0	4	32	0.485	0.486
T3N0M0	11	62	0.004	0.985
T2N1M0	10	50	0.163	0.686
T3N1M0	10	52	0.078	0.780
T4N2M0	6	20	1.457	0.227
T2N2M1	2	9	0.091	0.763

Histological type				
Squamous cell carcinoma	30	162	0.163	0.686
Adenocarcinoma	12	73	0.072	0.788
Undifferentiated carcinoma	3	20	0.075	0.784

Tumor location				
Upper esophagus	12	70	0.012	0.913
Median esophagus	30	165	0.065	0.799
Lower esophagus	3	20	0.075	0.784

**Table 2:** Analysis of the surgical factors.

Group	Occurrence group (*n* = 45)	Nonoccurrence group (*n* = 255)	*X* ^2^/*t*	*P*
Length of the resected esophagus (cm)	27.10 ± 5.23	24.23 ± 2.22	6.184	<0.001
Gastric tube reconstruction	15	175	20.518	<0.001
Whole stomach reconstruction	30	80	20.518	<0.001
Surgery time (min)	289.62 ± 9.67	264.58 ± 9.78	15.861	<0.001
Intraoperative blood loss (ml)	280.65 ± 9.65	262.35 ± 9.98	11.395	<0.001
Days of the gastrointestinal decompression (days)	7.00 ± 0.30	6.89 ± 0.38	1.842	0.066
Gastrointestinal decompression volume (ml)	2112.65 ± 9.65	2098.65 ± 9.98	8.718	<0.001

**Table 3:** Multivariate analysis of the reflux esophagitis in patients undergoing esophageal cancer surgery.

Factors	B	Wald	*P*	Exp (B)
Body weight	0.155	1.077	0.299	1.168
BMI	0.144	0.139	0.710	1.155
Length of the resected esophagus	−0.381	5.333	0.021	0.683
Whole stomach reconstruction	1.213	16.985	0.004	2.214
Intraoperative blood loss	−0.198	11.845	<0.001	0.821
Surgery time	−0.255	13.941	<0.001	0.775
Gastrointestinal decompression volume	−0.068	1.721	0.190	0.935

## Data Availability

The data used to support the findings of this study are available from the corresponding author upon request.
